# First-line single-agent regorafenib in frail patients with metastatic colorectal cancer: a pilot phase II study of the Spanish Cooperative Group for the Treatment of Digestive Tumours (TTD)

**DOI:** 10.1186/s12885-019-5753-7

**Published:** 2019-06-03

**Authors:** A. Carrato, M. Benavides, B. Massutí, R. Ferreiro-Monteagudo, P. García Alfonso, E. Falcó, M. Reboredo, T. Cano, J. Gallego, J. M. Viéitez, L. Layos, A. Salud, E. Polo, E. Dotor, G. Durán-Ogalla, M. Rodriguez-Garrote, A. Calvo, E. Grande, E. Aranda

**Affiliations:** 1 Medical Oncology Department, Hospital Universitario Ramón y Cajal, IRYCIS, CIBERONC, Alcala University, Ctra. De Colmenar Viejo, km 9,100, 28034 Madrid, Spain; 2 Hospital Regional Universitario Virgen de la Victoria, Málaga, Spain; 3 Hospital General Universitario de Alicante, Alicante, Spain; 4 Hospital Gregorio Marañón, Madrid, Spain; 5 Hospital Son Llatzer, Mallorca, Spain; 6 Complejo Hospitalario Universitario A Coruña, La Coruña, Spain; 7 Hospital Universitario Reina Sofia, IMIBIC, University of Córdoba, CIBERONC, Instituto de Salud Carlos III, Córdoba, Spain; 8 Hospital General Universitario de Elche, Alicante, Spain; 9 Hospital Universitario Central de Asturias, Oviedo, Spain; 10 Hospital Germans Trias i Pujol, ICO, Badalona, Spain; 11 Hospital de Lleida Arnau de Vilanova, Lérida, Spain; 12 Hospital Miguel Servet, Zaragoza, Spain; 13 Corporació Sanitària Parc Taulí, Barcelona, Spain

**Keywords:** Regorafenib, Colorectal cancer, Monotherapy, First-line, Frail patients, Elderly

## Abstract

**Background:**

Treatment of frail patients with advanced colorectal cancer (CRC) is controversial. This pilot phase II trial aimed to assess the efficacy and safety of regorafenib when administered in first-line to frail patients with advanced CRC.

**Methods:**

Frail patients without prior advanced colorectal cancer treatment were included in the study. Definition of frailty was defined per protocol based on dependency criteria, presence of chronic comorbid pathologies and/or geriatric features. Main objective: to assess progression-free survival (PFS) rate at 6 months. Treatment consisted of 28-day cycles of orally administered regorafenib 160 mg/day (3 weeks followed by 1 week rest).

**Results:**

Forty-seven patients were included in the study. Median age was 81 years (range 63–89). Frailty criteria: dependency was observed in 26 patients (55%), comorbidities in 27 (57%) and geriatric features in 18 (38%). PFS rate at 6 months was 45% (95% confidence interval [CI] 30–60]. Median PFS was 5.6 months (95%CI 2.7–8.4). Median overall survival (OS) was 16 months (95%CI 7.8–24). Complete response, partial response and stable disease were observed in one, two and 21 patients respectively (objective response rate 6.4%; disease control rate 51%). Thirty-nine patients (83%) experienced grade 3–4 adverse events (AEs). The most common grade 3–4 AEs were hypertension (15 patients; 32%), asthenia (14; 30%), hypophosphatemia (6; 13%); diarrhea (4; 8%), hand-foot-skin reaction (4; 8%). There were two toxic deaths (4.2%) (grade 5 rectal bleeding and death not further specified). Dose reduction was required in 26 patients (55%) and dose-delays in 13 patients (28%).

**Conclusions:**

The study did not meet the pre-specified boundary of 55% PFS rate at 6 months. Toxicity observed (83% patients experienced grade 3 and 4 AEs) preclude its current use in clinical practice on this setting. Disease control rate and overall survival results are interesting and might warrant further investigation to identify those who benefit from this approach.

**Trial registration:**

This trial was prospectively registered at EudraCT (2013–000236-94). Date of trial registration: April 9th, 2013.

## Background

CRC is the third most common cancer diagnosis after lung and breast cancer [1]. About 20% of patients with CRC have metastatic disease at diagnosis [2, 3] and up to 50% will have metastases at some point of the disease [2]. Median age at diagnosis of patients with CRC is 71. Therefore, a significant percentage of these patients are elderly and may be frail, due to either their age itself or comorbid conditions, leading to special vulnerability to treatment toxicity. Thus, the group of metastatic CRC patients who are frail comprises a mixture of elderly-frail patients, frail-non-elderly patients and very old patients who may be frail without any specific debilitating illness [4]. A chronologic transitional sequence “pre-frail to frail” state with a strong biological background has been advocated [5]. However, there is little consensus on the definition of frail patients and the limits between the terms elderly-frail-unfit. A few factors such as ageing, dependence for performance of daily activities, associated comorbid conditions, and presence of geriatric features (dementia, delirium, frequent falls, incontinence) are the most important to be taken into account for the definition of frailty [6].

Treatment of frail and/or elderly patients with advanced cancer is controversial. Systemic antineoplastic treatment, although well intentioned, may be too toxic leading to deterioration of frail cancer patients. These patients are commonly either totally excluded from participation or underrepresented in large pivotal clinical trials. Thus, the level of scientific evidence is generally low in this clinical setting and a more speculative approach is unavoidable for making treatment decisions. Outcomes achieved with chemotherapy in these patients with CRC have previously been addressed. Indeed, a randomized clinical trial in elderly and/or frail patients with metastatic CRC showed that treatment with single agent fluoropyrimidines resulted in similar efficacy outcomes and better quality of life, as compared with combination oxaliplatin-based chemotherapy [7]. In turn, irinotecan-based combination chemotherapy did not show advantage in terms of progression-free survival (PFS) over fluoropyrimidines alone in elderly patients [8]. Therefore, the appropriateness of polychemotherapy to treat these patients is controversial, and better tolerated regimens such as single agent regimens or new targeted drugs may be more suitable for treating frail patients.

Regorafenib (BAY 73–4506, Stivarga® Bayer HealthCare Pharmaceuticals Inc) is an oral multitargeted multikinase inhibitor with dual antiproliferative and antiangiogenic activity. A number of receptors such as VEFGFR1/3, KIT, TIE-2, PDGFR-β, FGFR-1, RET, RAF1 and B-RAF are the main targets for regorafenib [9, 10], which is approved for the treatment of advanced gastrointestinal stromal tumor (after sequential failure to front-line imatinib and second-line sunitinib) and pretreated metastatic CRC (after exposure to fluoropyrimidines, anti-VEGF therapy and anti-EGFR therapy if RAS wild type). Results from the CORRECT randomized study [11] showed that, as compared with placebo, regorafenib prolonged OS in patients with CRC previously treated with all approved standard therapies (6.4 versus 5.0 months; hazard ratio [HR] 0.77; 95% confidence interval [95% CI] 0.64–0.94; one-sided p 0.0052). Treatment was well tolerated being hand-foot skin reaction (HFSR), fatigue and hypertension the most frequent grade 3 or higher adverse events (AEs).

As the CORRECT study showed activity and manageable toxicity for regorafenib single agent, it was reasonable to investigate this strategy in first-line treatment of frail patients. Based on this background, this clinical trial was designed aiming to assess the efficacy and safety of regorafenib as a single agent in patients with metastatic CRC who were frail or unfit for chemotherapy.

## Methods

### Design

This study was designed as an open-label single-arm pilot phase II clinical trial. The study was approved by the Spanish Medicines Agency, by the Regional Clinical Research Ethics Committee of the Community of Madrid and was performed in accordance with the Good Clinical Practice guidelines and the last version of the Declaration of Helsinki (Fortaleza 2013). All patients provided written informed consent before enrolment.

### Patients and treatment

Patients older than 18 with histologically or cytologically proven advanced colorectal adenocarcinoma, without major surgery within 28 days prior to the initiation of study treatment, not previously treated for advanced disease, with measurable disease according to Response Evaluation Criteria In Solid Tumors (RECIST) v1.1, and an Eastern Cooperative Oncology Group (ECOG) performance status (PS) ≤ 2, were candidates to be enrolled in the study. Patients must have been frail and/or not candidates to receive combination chemotherapy as defined by the presence of one or more of the three criteria (a, b, c) as listed in Table 1. In addition, patients should have adequate organ function, as defined for bone marrow (absolute neutrophil count [ANC] > 1500/mm^3^; platelets > 100,000/mm^3^; hemoglobin > 9 g/dL), renal (creatinine clearance > 30 ml/min) and liver (bilirubin < 2.5 times x upper limit of normal [ULN], alanine aminotransferase [ALT] and aspartate aminotransferase [AST] < 3 x ULN or < 5 x ULN if liver metastases were present).

**Table 1:** Frailty criteria

a)	Dependency for daily activities due to comorbidities, different to deterioration from cancer.
b)	Previous history of three or more of these comorbidities, even under control because of a correct treatment:
	□ Congestive heart failure
	□ Other chronic cardiovascular diseases
	□ Chronic obstructive pulmonary disease
	□ Cerebrovascular disease
	□ Peripheral neuropathy
	□ Chronic renal failure^a^
	□ Arterial hypertension
	□ Diabetes mellitus
	□ Systemic vasculitis
	□ Severe arthritis
c)	At least one of these geriatric features:
	□ Age > 85 years
	□ Fecal or urinary incontinence
	□ Spontaneous bone fractures
	□ Mild or moderate dementia
	□ Frequent falls

Patients must be frail and/or not candidates to receive polychemotherapy as defined by the presence of one or more of the three criteria (a, b, c). ^a^However creatinine clearance should be > 30 mL/min for regorafenib treatment

Regorafenib single agent was administered at a dose of 160 mg/day (four 40 mg tablets) once a day by mouth, during 21 consecutive days followed by 7 days of rest. This 3 + 1 week schedule makes up a 28-day cycle. Regorafenib had to be taken in the morning, with some water after a light breakfast. Treatment was maintained until disease progression or unacceptable toxicity, physician discretion or patient decision for any reason. Dose modifications were performed in accordance with the Spanish product label. In summary, for administration of the next cycle, recovery of ANC to 1500/mm^3^ and platelets to 100,000/mm^3^ and recovery of the non-hematologic toxicities to National Cancer Institute Common Terminology Criteria (NCI-CTC) grade ≤ 2 were required. Grade 3–4 AEs led to a dose reduction except grade 4 hypertension, which led to permanent discontinuation. Three dose levels were established (160 mg/day, 120 mg/day and 80 mg/day) to make possible dose adjustments. Special management was required for HFSR, which should have recovered to grade ≤ 1 before resuming regorafenib and grade 2 or higher led to dose reduction.

### Study procedures

Progression was the main event for calculating the majority of the time to event variables of the study. This event in particular, and tumor response in general, was assessed according to RECIST v1.1 by the investigators. Image tumor assessments were performed every 8 ± 2 weeks. Both physical exam with blood pressure measurement and blood analysis (complete blood count, liver function tests, creatinine, albumin, glucose, urea and phosphorus) were performed weekly during the first two cycles and every other week thereafter. Assessment of carcinoembryonic antigen (CEA) was performed every cycle and test-strip monitoring for proteinuria every two cycles (if positive, a 24 h urine sample assessment was mandatory). The AEs were graded according to the NCI-CTC v4.0.

### Statistical analysis

We considered that a 55% PFS rate at 6 months would be a clinically relevant outcome with regorafenib treatment. Sample size calculation showed that 46 patients were required to both establish this PFS rate at 6 months and to reject the null hypothesis (defined as a PFS rate lower than 35%), with an alpha error of 0.05 and 80% power. The intention to treat (ITT) population was the analysis set and included all patients enrolled in the study who received at least one cycle of treatment and had at least one efficacy or safety evaluation.

The statistical analyses of the primary objective (PFS rate at 6 months) as well as the other time to event variables (duration of response, OS, time to response, time to progression, and treatment failure) were performed by the Kaplan-Meier product limit method. Tumor response (and other qualitative variables) were described with frequencies and percentages whereas quantitative variables were described with mean and/or median and range.

## Results

### Patient characteristics

Fifty-five patients were screened and 47 were included in the study between June 2013 and February 2015 in 13 hospitals in Spain. These patients were part of both the ITT population and the safety population. Table 2 summarizes baseline characteristics of patients. Briefly, median age was 81 years (range 63–89) and 21 patients (45%) were female. Thirty patients (64%) had an ECOG-PS 0–1 and 15 patients (32%) had a primary rectal adenocarcinoma. The most frequent sites of metastases were liver in 31 patients (66%) and lung in 29 patients (62%). Thirty-one patients (66%) had previous surgery for the primary colorectal tumor and seven patients (15%) received previous adjuvant chemotherapy (four patients had capecitabine single agent and three oxaliplatin plus capecitabine). Seventeen patients (36%) had only one organ involved by metastatic disease. Regarding the frailty criteria, dependency was observed in 26 patients (55%), comorbidities in 27 (57%) and geriatric features in 18 (38%). Twenty patients (42%) fulfilled a combination of two or three frailty criteria.

**Table 2:** Patient characteristics and exposure to regorafenib treatment

	*N* = 47
Gender, n %	
Male	26 (55)
Female	21 (45)
Age (years), median [range]	81 [63–89]
ECOG PS, n %	
0	5 (11)
1	25 (56)
2	17 (36)
Frailty criteria, n %	
Dependence for daily activities	8 (17)
History of comorbidities	13 (28)
Geriatric symptoms	6 (13)
Dependence + Comorbidities	8 (17)
Dependence + Geriatric features	6 (13)
Comorbidities + Geriatric Features	2 (4.3)
Dependence + Geriatric Features + Comorbidities	4 (8.5)
Primary tumor site, n %	
Colon	32 (68)
Rectum	14 (30)
Both	1 (2.1)
Metastatic at first diagnosis, n %	30 (64)
Metastatic sites, n %	
Liver	31 (66)
Lung	29 (62)
Peritoneum	11 (23)
Bone	1 (2.1)
Number of organs involved by M1 disease, n %	
1	17 (36)
2	14 (30)
3	12 (25)
4	2 (4.3)
5	2 (4.3)
Prior surgery, n %	31 (66)
Prior radiation therapy, n %	6 (13)
Prior adjuvant chemotherapy, n %	7 (15)
Capecitabine alone	4 (0.8)
Capecitabine-oxaliplatin	3 (0.6)
Exposure to regorafenib	
Dose intensity (mg/day), median [range]	91 [58–121]
Relative dose intensity (mg/day/theoretical total dose), % [range]	0.76 [0.48–1.01]

### Efficacy and dose modifications

Median follow-up was 10.7 months. PFS rate at 6 months was 45% (95%CI 30–60) (Fig. 1). Median PFS was 5.6 months (95%CI 2.7–8.4) (Table 3). Median OS was 16 months (95%CI 7.8–24) (Fig. 1). Response was not evaluable in 10 patients who discontinued before first scheduled radiological assessment (4 patients due to AEs, 4 patient decision and 2 toxic deaths).

**Fig. 1:** Progression free survival and Overall survival

**Table 3:** Efficacy results

	ITT population (*N* = 47)
Best objective response	
Overall response rate, %	6.4
Complete response, n (%)	1 (2.1)
Partial response, n (%)	2 (4.3)
Stable disease, n (%)	21 (45)
Progression disease, n (%)	13 (28)
Disease control rate, n %	24 (51)
Non-evaluable, n %	10 (21)
Progression free survival (months), median (95%CI)	5.6 (2.7–8.4)
Progression free survival, rate at 6 months (95%CI)	45% (30–60)
Overall survival (months), median (95%CI)	16 (7.8–24)
Time to treatment failure (months), median (95%CI)	2.1 (1.3–2.9)
Time to progression (months), median (95%CI)	5.6 (1.9–9.3)

*N = 21 for stable disease analysis; Disease control rate = Overall response rate + stable disease rate

Complete response and partial response were observed in one and two patients, respectively, leading to 6.4% objective response rate in the ITT population. Stable disease was observed in 21 patients leading to 51% disease control rate. Response assessment was investigator-based and not centrally reviewed.

A total of 198 cycles of regorafenib (3 weeks of each 4 week cycle) were administered to 47 patients (mean 4.2 cycles, median 2.0 and range 1–20), and 23 cycles had to be delayed (12%). Thirteen patients (28%) required one to four delays. The most common cause of delay was non-hematologic toxicity (asthenia in 3 cycles, urinary tract infection in 3 cycles and diarrhea in 2 cycles). Dose reduction was required in 26 patients (55%) who needed one (16 out of 26 patients; 61%) or two dose reductions per patient. The most common cause of dose reduction was fatigue (12 out 37 cycles; 32%) followed by HFSR and mucositis (4 cycles each; 11%); hypophosphatemia and hypertension (2 cycles each; 5.4%). Median relative dose intensity (mg/day/planned total dose) was 76% (range 48–101). Among the patients with complete and partial response, all of them necessitated dose reduction (only one patient needed two dose reductions), one of them required dose delays (3 cycles delayed: one for asthenia and two for administrative reasons), and the relative dose intensity among these patients ranged between 83 and 62%.

### Safety and post-study treatments

Thirty-nine patients (83%) experienced grade 3–4 AEs. The most common grade 3–4 AEs were hypertension (15 patients; 32%), asthenia (14; 30%), hypophosphatemia (6; 13%); diarrhea (4; 8%), HFSR (4; 8%), increased AST (3; 6.4%), mucositis 3 (6.4%) (Table 4). Other grade 3–4 AEs occurred in less than 5% of patients. Grade 3–4 AEs were observed in 101 out of 198 cycles administered (51%), mainly in the first two cycles. Twenty-two patients (47%) experienced serious AEs (SAEs). Among them, 13 patients (28%) experienced regorafenib-related SAEs. Eleven patients (23%) discontinued treatment because of toxicity being the most frequent fatigue. Besides toxicity, the reason for regorafenib treatment withdrawal was death in three patients (6.4%), intercurrent disease/AE not related to the treatment in four patients (8.5%), decision of the patient/investigator in 11 patients (23%), and disease progression in 18 patients (38%). There were two drug-related deaths. A fatal rectal primary tumor bleeding occurred during the first cycle at a regorafenib dose of 160 mg/day in an 86-year-old patient. The family decided palliative care and did not authorize blood transfusions or an invasive approach. The second event was reported in an 84-year-old patient who suffered a sudden death at home when sleeping, being asymptomatic the previous day, during the second cycle at a regorafenib dose of 160 mg/day.

**Table 4:** Grade 3–5 adverse events related to regorafenib

Adverse event	Grade 3 *n* (%)	Grade 4 *n* (%)	Grade 5 *n* (%)	Total (Grade3–5) *n* %
Hypertension	14 (30)	1 (2.1)	0	15 (32)^a^
Fatigue	14 (30)	0		14 (30)
Hypophosphatemia	6 (13)	0	0	6 (13)
HFSR^a^	4 (8.5)	0	0	4 (8.5)
Diarrhea	4 (8.5)	0	0	4 (8.5)
Increased AST	3 (6.4)	0	0	3 (6.4)
Increased GGT	3 (6.4)	0	0	3 (6.4)
Mucositis	3 (6.4)	0	0	3 (6.4)
Anorexia	2 (4.3)	0	0	2 (4.3)
Increased bilirubin	2 (4.3)	0	0	2 (4.3)
Increased lipase	1 (2.1)	1 (2.1)	0	2 (4.3)
Rectal bleeding	1 (2.1)	0	1 (2.1)	2 (4.3)
Hyperuricemia	0	1 (2.1)	0	1 (2.1)
Sudden death	0	0	1 (2.1)	1 (2.1)
Stroke	1 (2.1)	0	0	1 (2.1)
Pancreatitis	1 (2.1)	0	0	1 (2.1)
Stomathitis	1 (2.1)	0	0	1 (2.1)
Hyperglucemia	1 (2.1)	0	0	1 (2.1)
Skin rash	1 (2.1)	0	0	1 (2.1)
Proteinuria	1 (2.1)	0	0	1 (2.1)
Pancreatitis	1 (2.1)	0	0	1 (2.1)
Nausea	1 (2.1)	0	0	1 (2.1)
Constipation	1 (2.1)	0	0	1 (2.1)
Vaginitis	1 (2.1)	0	0	1 (2.1)
Aphonia	1 (2.1)	0	0	1 (2.1)
Somnolence	1 (2.1)	0	0	1 (2.1)
Dry mouth	1 (2.1)	0	0	1 (2.1)
Abdominal pain	1 (2.1)	0	0	1 (2.1)
Increased ALT	1 (2.1)	0	0	1 (2.1)
Tumor abscess	1 (2.1)	0	0	1 (2.1)
Pneumonia	1 (2.1)	0	0	1 (2.1)
Intestinal perforation	1 (2.1)	0	0	1 (2.1)

^a^12 out 15 patients (89%) who experienced hypertension, presented hypertension at baseline

*Abbreviations*: *HFSR* Hand Foot Skin Reaction

Nineteen patients (40%) received second and further lines of therapy after study treatment discontinuation. The majority received single agent fluropyrimidine-based treatment. One of the patients treated with capecitabine also had complete resection of liver metastases. Two patients received capecitabine-oxaliplatin and one of them was further treated with panitumumab-irinotecan. Another patient received capecitabine-bevacizumab. The range of the number of post study lines was [1-5] and only two patients received more than two lines after regorafenib (one received 3 single-agent treatments and the other one received 5 single-agent treatments).

## Discussion

This study shows that, when treated with frontline regorafenib, almost half of frail patients with advanced CRC remain PFS at 6 months and that this treatment resulted in 16 months median OS. Although the study did not meet the pre-specified boundary of 55% PFS rate at 6 months, median overall survival is remarkable high when compared with other biologic agents in the same setting. Indeed, panitumumab resulted in median OS of 12.3 months in a population of frail-elderly patients with wild-type KRAS tumors [12]. Cetuximab resulted in 11.1 months of median OS in elderly-fit patients [13]. Addition of capecitabine to cetuximab resulted in improved outcomes (median OS 16.1 months) with a higher skin toxicity, mostly paronychia [14]. Yet, it should be mentioned that the OS might be affected by the subsequent treatment lines, and in this study, 40% of patients received chemotherapy after regorafenib. In addition, regorafenib resulted in 5.6 months median PFS which compares favorably with other single agent regimens such as 5-fluorouracil (3.5 months) [7], panitumumab (4.3 months in KRAS wild-type) or cetuximab (2.9 months in RAS non-selected) [13] but seems to be inferior to doublets such as cetuximab-capecitabine (8.4 months in KRAS wild-type) [14] or bevacizumab-capecitabine (9.1 months) [15]. Regorafenib, like many targeted tyrosine-kinase inhibitors, lacks at this moment a specific biomarker [16].

Other different strategies have been addressed in frail and/or elderly patients. Comparing with fluoropyrimidines-based chemotherapy, OS with regorafenib in our trial is clearly longer than the approximately 11 months achieved with fluoropyrimidines (either 5-fluorouracil or capecitabine) with or without oxaliplatin in the FOCUS 2 trial [7]. Our OS is in line with results of bevacizumab with capecitabine combination as shown in the AVEX randomized trial, which compared capecitabine-bevacizumab versus capecitabine alone resulting in a non-significant difference of 20 versus 16 months in median OS [15]. However, an important difference should be mentioned on the definition of frailty, which was left to investigator discretion in the AVEX trial whereas it was strictly predefined in our study. Response rate was low in our trial, as expected, because this is what is commonly observed with the use of new kinase inhibitors [17]. However, a disease control rate of 51% should be underlined because the clinical value of disease stabilization is a relevant outcome in metastatic CRC [18]. Furthermore, this benefit may be more valuable in the group of frail patients due to the fact that, frailty itself has shown to be an independent factor associated with poor prognosis in older patients with CRC [19].

After the initiation of our study, two additional trials performed on similar but pretreated patient population with CRC, contributed to expanding safety information available from the CORRECT trial [11]. The REBECCA study was a phase IV clinical trial [20] and the CONCUR study was a randomized trial conducted in Asia with the same design as the CORRECT study [21]. Altogether, these three trials have defined the pattern of toxicity of regorafenib with HFSR, hypertension, fatigue and hypophosphatemia being the most frequent AEs. Our results are in line and show that the safety results should be put into perspective (i.e. comorbidities, etc.) when administered in frontline to frail patients. Like in other studies [11, 20–23] the percentage of patients who experienced grade 3 or higher AEs is high, mainly in the first cycle, but preventable for further cycles by performing dose modifications. This makes it easier for regorafenib continuation, thus allowing the patients to obtain the benefits from the treatment [24]. Indeed, in our study, this idea is clearly underlined by the fact that rate of grade 3 or higher AEs decreases from 83%, when calculated by patient, to 51% when calculated by cycle. The rate of SAEs we observed (47%) is higher than that in the CORRECT phase II trial (43%) and substantially higher than the rate of treatment-related SAEs (27%). This may be due to the nature of a frail population, which may lead to a need of hospitalization from an AE, in a patient who otherwise should not need it. We had already observed in our previous study of frontline panitumumab in elderly-frail patients a 36% SAEs rate [12] which is higher than that expected for panitumumab single agent. The overall safety profile we observed calls for a recommendation taking into account that an appropriate familial and social support is needed in order to prescribe a treatment with regorafenib in a frail patient. A close monitoring of patients under treatment is also needed. For the same reason, an initial treatment dose of 120 mg daily is a reasonable approach with the possibility of escalating if no SAEs and toxicities are observed. A randomized phase 2 study is being conducting to compare different dose approaches of induction treatment (first cycle) of regorafenib in metastatic CRC patients. ClinicalTrials.gov identifier: NCT02835924 [25].

The present study has some limitations. First, firm conclusions cannot be drawn from a small, single-arm study and the results should be confirmed in further larger trials. Second, this study has not an associated pharmacoeconomic study, which may be a concern when an innovative and costly treatment is being administered to frail and/or elderly patients who have competing causes of death. Third, the absence of a standardized definition of frailty makes it hard to carry out inter-study comparisons. Unfortunately, heterogeneity is very frequent in the studies conducted in this field, which are being performed on several different types of patients with or without some, but not all, characteristics of frailty-elderly-unfit. And fourth, not assessing of quality of life.

## Conclusions

In conclusion, the study did not meet the pre-specified boundary of 55% PFS rate at 6 months. However, after considering the results of the panitumumab study in frail patients [12] published in 2015, when the present study was ongoing, our pre-determined boundary might be considered too optimistic. Results on disease control rate and OS provided by regorafenib single agent in this study are interesting and might warrant further investigation to identify those patients who benefit from this approach. A higher incidence of grade 3–4 AEs rate as well as regorafenib dose-reduction and delays rates preclude its current use in clinical practice on this setting. This suggests that the most appropriate initial dosing approach for this patient population should be evaluated further, as well as to define more accurately the subgroup of frail patients who may derive the maximal benefit and those patients with an excessive risk of toxicity [26]. Investigation on biomarkers must be helpful in order to achieve these goals.

## Data Availability

The datasets used and/or analyzed during the current study are available from the corresponding author on reasonable request.

## Abbreviations

AE: Adverse event
ALT: Alanine aminotransferase
ANC: Absolute neutrophil count
AST: Aspartate aminotransferase
CEA: Carcinoembryonic antigen
CRC: Colorectal cancer
ECOG: Eastern cooperative oncology group
HFSR: Hand-foot skin reaction
HR: Hazard ratio
ITT: Intention-to-treat
NCI-CTC: National cancer institute common terminology criteria
PFS: Progression-free survival
PS: Performance status
SAE: Serious Adverse Event
RECIST: Response evaluation criteria in solid tumors
ULN: Upper limit of normal
95%CI: 95% confidence interval
